The article "Experimental Study on Danggui Shaoyao San Improving Renal Fibrosis by Promoting Autophagy" was published in 2022. Journal: Evid Based Complement Alternat Med.

# Experimental Study on Danggui Shaoyao San Improving Renal Fibrosis by Promoting Autophagy

**DOI:** 10.1155/2022/6761453

**Published:** 2022-07-31

**Authors:** Lian Fan, Hui-hua Chen, Hua-jun Liu, Hui-juan Chen, Ling-ling Zhu, Ting Zhang

**Affiliations:** The Teaching and Research Office for Fundamentals of Traditional Chinese Medicine, Shanghai University of Traditional Chinese Medicine, 1200 Cailun Road, Shanghai 201203, China

## Abstract

Renal fibrosis could lead to chronic kidney disease (CKD) developing into the end-stage with its pathological manifestation is the deposition of extracellular matrix (ECM). Danggui Shaoyao San (DSS) is one of the widely used herbal formulas in ancient China, which has been proven to have efficacy in the treatment of CKD. The experiment employed TGF-*β*1 to stimulate the NRK-52E cells to establish a renal fibrosis model. With rapamycin (RAPA) used as the positive control, we detected the expression of fibronectin (FN), caspase-3, and autophagy-related proteins in the NRK-52E cells treated with DSS by Western blot and immunofluorescence assay. In order to further verify autophagy-promoting effects of DSS, we adopted 3-MA to inhibit autophagy. The experiment has found that DSS can lower the protein levels of FN and caspase-3 in the NRK-52E cells induced by TGF-*β*1. After TGF-*β*1 stimulation, the expression of LC3 II/I and Beclin 1 has decreased, and the protein levels of mTOR and p62 have increased. Consistent with rapamycin, DSS has significantly reduced these effects of TGF-*β*1. It has also been found that DSS can increase the expression of LC3 II/I and Beclin 1 proteins and can reduce the level of mTOR in cells treated with 3-MA, suggesting that DSS can promote autophagy. In conclusion, DSS has been proved to reduce the apoptosis and fibrosis of NRK-52E cells induced by TGF-*β*1, which may be achieved by promoting autophagy.

## 1. Introduction

In recent years, chronic kidney disease (CKD) has become one of the major global public health problems due to its high incidence [1]. Renal fibrosis is the common pathway of all CKD developing into the end-stage, and its pathological manifestation is the deposition of fibrous matrix such as collagen, fibronectin, and laminin in renal tubules and surrounding capillary spaces caused by various stimulating factors. Excessive deposition of the extracellular matrix (ECM) may cause renal dysfunction, which leads to renal fibrosis and ultimately renal failure. At present, a large number of studies have shown that there is a certain correlation between the progression of renal fibrosis and autophagy [2, 3]. Autophagy refers to a catabolic process in which lysosomes are used to degrade damaged and aging biological macromolecules and organelles, so that cells can digest and recover cytoplasmic components, which plays an important role in maintaining normal physiological activities [4]. Autophagy in mammalian cells can be induced by starvation or drugs such as rapamycin, while drugs including 3-methyladenine (3-MA) and chloroquine can inhibit autophagy [5]. In CKD, a variety of proteins have been proved to alleviate kidney damage, such as antiaging protein Klotho, uncoupling protein 2, and lactoferrin, whose mechanism of action depends on the function of promoting autophagy [6–8]. Atg5-mediated autophagy in proximal renal tubular epithelial cells (TECs) ameliorates renal fibrosis by reducing G2/M cell cycle arrest and inflammatory cell infiltration and cytokine production [9]. However, another study found that autophagy induced by the transcription factor EB can mediate the apoptosis of TECs, thereby aggravating the progression of renal fibrosis [10]. In a rat model of renal fibrosis following unilateral ureteral ligation (UUO), downregulation of autophagy alleviates disease progression [11]. The mechanisms of autophagy involved in renal fibrosis are complex, but it is certainly an attractive target in the search for therapeutic approaches to CKD.

Danggui Shaoyao San (DSS) was originally recorded in *Synopsis of Prescriptions of the Golden Chamber (Jīn Guì Yào Lüè)*, written by Zhongjing Zhang in the Eastern Han Dynasty (25–220). The ingredients in this formula include Danggui, Baishao, Chuanxiong, Fuling, Baizhu, and Zexie. DSS was mainly used for the treatment of edema and gynecological miscellaneous diseases in ancient times. In modern times, it is often adopted to treat diseases such as CKD, Alzheimer's disease, primary dysmenorrhea, and depression with good clinical efficacy [12–14]. Experiments have shown that DSS can reduce renal tubule epithelial-mesenchymal transformation (EMT) by inhibiting the Notch signaling pathway, thereby improving renal fibrosis and preventing diabetic nephropathy [15]. In our previous studies, we found that DSS can protect the kidney via alleviating tissue hypoxia and reducing renal hypertrophy and renal dysfunction induced by UUO. In this experiment, we also found that after DSS intervention, the level of LC3 II/I in renal tissues was increased and the expression of p62 protein was downregulated, suggesting that DSS may play a role in promoting autophagy [16]. The purpose of this study was to investigate the autophagy-inducing effect of DSS on the TGF-*β* 1-induced NRK-52E cells' renal fibrosis model, so as to study the mechanism of related treatment mediated by DSS.

## 2. Materials and Methods

### 2.1. Preparation of DSS

DSS is composed of Danggui, Baishao, Chuanxiong, Fuling, Baizhu, and Zexie in a dry weight ratio of 10 : 30 : 9:20 : 20 : 15. All the ingredients were supplied by the Shanghai Lei Yun Shang West Pharmaceutical Retail Co., Ltd. (Shanghai, China) (Table 1). Aqueous DSS was diluted 10 times in distilled water and heated at 100°C for 3 h under a continuous stirring condition. After filtering, the residue was diluted 8 times in distilled water and repeatedly heated at 100°C for 3 h under a continuous stirring condition. The mixed extract was subjected to centrifugation at 1500 × *g*. The supernatants were collected and kept under low temperature at −70°C for evaporation until semisolid state of DSS (lyophilized powder) is formed. When using, it can be directly diluted to the desired concentration with a serum-free medium.

### 2.2. Cell Culture and Treatment

The NRK-52E cell line was purchased from Shanghai Enzyme Research Biotechnology Co., LTD. (Shanghai, China), in a DMEM high sugar culture medium (Gibco, NY, USA) containing 10% fetal bovine serum (FBS; Every Green, Hangzhou, China) and 100 U/ml penicillin-streptomycin (Gibco, NY, USA). Cells were incubated at 37°C and 5% CO2. Group intervention: The blank control group was cultured in a serum-free DMEM medium, and the model group was stimulated with 5 ng/ml TGF-*β*1 (PeproTech, NJ, USA). The treatment group was incubated with DSS and the positive drug control group was incubated with 10 nM rapamycin (Sangon Biotech, Shanghai, China) for 48 h on the basis of the model group. In order to further study the therapeutic effect of DSS, the cells were divided into the following groups: The blank control group was cultured in a serum-free DMEM medium, the autophagy-inhibited group was stimulated with 10 mM 3-MA (MCE, Shanghai, China), and the treatment group was incubated with 10 mM 3-MA + 0.8 mg/ml DSS for 24 hours.

### 2.3. Cell Survival Assay

The CCK-8 assay was conducted to evaluate the survival of NRK-52E cells upon TGF-*β*1 and DSS treatment as described. Cells were plated into 96-well plates at a density of 1∼1.5 × 10^4 cells per well. Ten microliters of the CCK-8 reagent (Beyotime, Shanghai, China) was added and incubated for 90 min. The optical density (OD) was measured using a microplate reader (BioTek, Vermont, USA) at 450 nm. The procedure was carried out thrice to obtain the mean values.

### 2.4. Western Blotting Analysis

Cellular protein lysates were separated by 10–12% SDS-PAGE and then transferred to PVDF. The membranes were probed overnight at 4°C with primary antibodies against fibronectin (Abcam, Cambridge, CB, UK), caspase-3(Abcam, Cambridge, CB, UK), Phospho-mTOR (CST, Danvers, MA, USA), mTOR (Abcam, Cambridge, CB, UK), Beclin 1(Abcam, Cambridge, CB, UK), LC3B (Abcam, Cambridge, CB, UK), p62(CST, Danvers, MA, USA), GAPDH (Proteintch, Rosemont, IL, USA), and *β*-actin (Proteintch, Rosemont, IL, USA). The next day, the membranes were washed and incubated with the appropriate secondary antibody for 1.5 h at room temperature. After the final wash, signals were detected using the FluorChem E imaging system (ProteinSimple, San Francisco, CA, USA) and a chemiluminescence detection kit (EMD Millipore). Protein band densities were quantified by using an image analysis system (Alpha View SA, ProteinSimple, San Francisco, CA, USA) and expressed as ratios to GAPDH or *β*-actin.

### 2.5. Immunofluorescent Staining

Cells were fixed with 4% paraformaldehyde for 20 min, permeabilized with 0.1% Triton X-100 for 15 min, blocked with 5% BSA for 1 h, and incubated overnight at 4°C with anti- LC3B (ab192890, Abcam, Cambridge, CB, UK). The cells were then incubated with ALexa Fluro® 488 conjugated anti-rabbit antibody (Beyotime, Shanghai, China) for 1.5 h at room temperature and stained with 4ʹ,6-diamidino-2-phenylindole (DAPI; Beyotime, Shanghai, China) for 15 min. Images were captured by laser confocal microscopy (ZEISS, Oberkochen, Germany).

### 2.6. Statistical Analysis

SPSS21.0 was adopted to analyze the data and results were presented as means ± SEM. Data from the experimental groups were compared by one-way analysis of variance (ANOVA) followed by Tukey's post hoc analysis; *p* < 0.05 indicated statistical significance.

## 3. Results

### 3.1. Selection of DSS Treatment Concentration

First, the cytotoxicity test of Danggui Shaoyao San was carried out. Under different stimulation times, different concentrations of DSS had different effects on NRK-52E cell activity (Figure 1(a)). Next, cells were stimulated with the drug concentration of DSS which has no significant cytotoxic effect at 5 ng/ml TGF-*β*1 for 48 h. Moreover, the results showed that the cell activity was above 80% (Figure 1(b)). Then, we chose the dosages 0.4, 0.8, and 1.6 mg/ml drug concentration of DSS to stimulate the NRK-52E cells for 48 h on the basis of model group. The WB results displayed that compared with the model group, after DSS intervention, LC3 II/I showed an increasing trend, while FN and caspase-3 showed a decreasing trend (Figures 1(c) and 1(d)). So, we chose the dosage 0.8 mg/ml drug concentration of DSS which could significantly decrease FN secretion, reduce apoptosis, and promote autophagy of NRK-52E cells induced by TGF-*β*1 as the final therapeutic concentration.

### 3.2. DSS Decreased FN Secretion and Apoptosis of NRK-52E Cells Induced by TGF-*β*1

In order to investigate whether DSS has a therapeutic effect on the cellular renal fibrosis model, the protein levels of FN, a marker of NRK-52E cells fibrosis, and caspase-3, an apoptosis-related factor, were detected after TGF-*β*1 treatment. The results showed that TGF-*β*1 induced the expression levels of FN and caspase-3 in the NRK-52E cells that were significantly increased, while DSS and rapamycin could significantly inhibit the increase of these proteins (Figure 2); thus, we believe that DSS has a certain therapeutic effect on renal fibrosis. In conclusion, DSS can reduce FN secretion and apoptosis of NRK-52E cells induced by TGF-*β*1.

### 3.3. DSS Promoted the Autophagy of NRK-52e Cells Induced by TGF-*β*1

In order to test whether DSS can regulate the autophagy of NRK-52E cells stimulated by TGF-*β*1, the protein expressions of the following autophagy markers were detected: LC3B, Beclin 1, mTOR, and p62. The results showed that after TGF-*β*1 stimulation, the expression of LC3 II/I and Beclin 1 decreased, and the protein levels of mTOR and p62 increased, while DSS upregulated the expression of LC3 II/I and Beclin 1, and decreased the levels of mTOR and p62. This is consistent with the results of the autophagy inducer rapamycin (Figures 3(a) and 3(b)), suggesting that DSS may increase the autophagy level of cells. In order to further compare the differences in autophagy among the groups, LC3B, one of the most representative proteins, was selected for immunofluorescence detection. The trend was the same as that of WB, and both DSS and rapamycin could inhibit the reduction of autophagy caused by TGF-*β*1 (Figures 3(c) and 3(d)). In conclusion, DSS can promote the autophagy of NRK-52E cells induced by TGF-*β*1.

### 3.4. DSS Can Suppress the Autophagy Inhibition of 3-MA

In order to further verify the autophagy promoting effect of DSS, the expression levels of LC3B, Beclin 1, mTOR, and other proteins in NRK-52E cells were detected under the intervention of autophagy inhibitor 3-MA. WB results showed that 3-MA significantly reduced intracellular LC3B and Beclin 1 protein levels and upregulated mTOR expression. DSS was able to inhibit these effects (Figure 4(a) and 4(b)). Immunofluorescence results suggested that intracellular autophagy flux decreased after 3-MA stimulation, while DSS significantly increased intracellular LC3B expression (Figure 4(c) and 4(d)). In conclusion, DSS can inhibit the autophagy inhibition of 3-MA and has the ability to promote autophagy.

## 4. Discussion

The incidence and prevalence of CKD have increased significantly worldwide. Currently, there is a lack of effective and targeted treatment drugs. A considerable number of cases will progress to end-stage renal failure, requiring lifelong dialysis or kidney transplantation [17]. Renal fibrosis is considered to be the common pathway of all forms of CKD. Therefore, it is urgent to find promising drugs to treat renal fibrosis. At present, it is believed that renal epithelial cells can undergo phenotypic transformation into myofibroblasts induced by some growth factors or inflammatory factors, which are the main source of extracellular matrix and play an important role in the occurrence and development of renal fibrosis [18]. Therefore, the NRK-52E cells were selected as experimental subjects to study renal fibrosis.

DSS is a commonly used classical formula in ancient times, mainly used for the treatment of gynecological diseases, but now there is a lot of evidence to prove that this formula also has advantages in the treatment of CKD [19, 20]. Studies have shown that total glucosides of paeony could retard the process of fibrosis and reduce the pathological damage in adriamycin-induced rats by downregulating the expression of TLR4/NF-*κ*B/TGF-*β*1 signaling [21]. Moreover, ligustrazine (LIG is a purified and chemically identified component of the Chinese herb Ligusticum wallichii Franchat) was found to improve renal interstitial fibrosis in UUO rats by reducing the mRNA expression of TGF-*β*1, CTGF, monocyte chemoattractant protein-1, and osteopontin [22]. Besides, Wang found that the treatment of DSS was probably related to the regulation of amino acid and energy metabolism using metabolic pathway analysis [20].

The excessive secretion of TGF-*β*1 is one of the direct factors leading to renal fibrosis [23, 24], that is why TGF-*β*1-stimulated cells was used to establish an in vitro model of renal fibrosis. The results showed that the level of fibronectin in the NRK-52E cells significantly increased after TGF-*β*1 stimulation, suggesting the occurrence of renal fibrosis, while the expression level of FN decreased after the dosages 0.8 and 1.6 mg/ml drug concentration of DSS treatment, suggesting that DSS can treat renal fibrosis. In addition, the effect of apoptosis on fibrosis cannot be ignored; inhibiting the apoptosis of renal tubular cells can prevent renal function injury and the development of fibrosis [25, 26]. As a typical apoptotic effector, caspase-3 has been confirmed to increase the injury of microvascular endothelial cells, cause cell death, and aggravate renal injury [27]. Our study showed that the dosages 0.4 and 0.8 mg/ml drug concentration of DSS could reduce the level of caspase-3 protein in the NRK-52E cells induced by TGF-*β*1, suggesting that DSS may improve renal fibrosis by reducing apoptosis. According to the expression results of FN and caspase-3 in model cells under different concentrations of DSS intervention, the dosage 0.8 mg/ml drug concentration of DSS was selected as the treatment concentration.

Autophagy is a cellular self-digestion mechanism that degrades damaged organelles and plays an important role in maintaining normal physiological activities of cells. When stimulated by certain autophagy-inducing factors, the ULK1 complex dissociates from mTORC1 and activates autophagy. After that, Atg6/Beclin 1 mediates the formation of an autophagy precursor membrane. LC3-II formed by Atg processes locates on the inner and outer membrane of autophagosome and participates in the extension of the double membrane structure of autophagy precursor, forming autophagosome and maturing [28, 29]. However, a large number of studies have shown that autophagy can participate in the occurrence and development of renal fibrosis through multiple pathways, including TGF-*β*/Smad4 signaling pathway, PI3K/Akt/mTOR signaling pathway, MEK/ERK/NRF-1 signaling pathway, and silencing regulatory protein 1(SIRT1)-mediated autophagy [30–33]. Our results showed that after TGF-*β*1 stimulation, the expression of LC3 II/I and Beclin 1 in the NRK-52E cells decreased, and the protein level of mTOR increased, indicating that autophagy was inhibited in the process of renal fibrosis, which was also confirmed by the increased expression of autophagy substrate p62. However, after DSS treatment, the expression of the above proteins showed an opposite result, which was consistent with the trend caused by the autophagy inducer rapamycin. Next, we used immunofluorescence to detect LC3B, which is widely used in the detection of autophagy because it locates directly on the autophagosome membrane, and found that DSS can significantly reduce the inhibition of autophagy caused by TGF-*β*1. In order to further verify the ability of DSS to promote autophagy, after 3-MA was used to inhibit autophagy, it was found that DSS still could significantly increase intracellular LC3 II/I and Beclin 1 protein levels, and reduce the expression of mTOR, suggesting that DSS can indeed promote autophagy.

Consistent with our results, many Chinese herbal extracts have been proved to inhibit renal fibrosis by increasing autophagy, reducing ECM accumulation and kidney damage [34–37]. However, some studies have found that the increase of autophagy can aggravate renal fibrosis. For example, Tang S et al. believe that TGF-*β* can promote autophagy by inhibiting the endogenous inhibitor of pro-fibrosis signaling pathway―Ptch1, thereby aggravating renal fibrosis [38]. Drugs such as l-carnitine have been shown to improve renal fibrosis by downregulating autophagy [11, 39]. These two opposite results may be caused by different drugs and different pathways of action, and there may be important cofactors between autophagy and renal fibrosis that need to be further explored. We will focus on other molecular mechanisms by which DSS improves renal fibrosis and explore its synergistic effect. Furthermore, in this study, we investigated the compound of DSS; in the future, we would explore the active ingredient of DSS to exert antirenal fibrosis by conducting a study at the system and omics levels.

In conclusion, this study proves that DSS can reduce the apoptosis and fibrosis of NRK-52E cells induced by TGF-*β*1, which may be achieved by promoting autophagy, but the mechanism should be executed for further research.

## Figures and Tables

**Figure 1:** Selection of DSS treatment concentration. (a) NRK-52E cells were treated, respectively, with different drug concentrations of DSS (0, 0.2, 0.4, 0.8, 1.6, 3.2, 6.4, and 12.8 mg/ml) for different time periods (24 h, 48 h, and 72 h) (*n* = 3, per group). (b) NRK-52E cells were treated, respectively, with different drug concentrations of DSS (0, 0.2, 0.4, 0.8, 1.6, and 3.2 mg/ml) at 5 ng/ml TGF-*β*1 for 48 h (*n* = 5, per group). Then, NRK-52E cells were treated, respectively, with 5 ng/ml TGF-*β*1 and different drug concentrations of DSS (*n* = 3, per group). “+” means containing the drug, “--” means without the reagent, “0.4, 0.8, 1.6” means the used drug concentration of DSS (mg/ml). (c) Protein levels of LC3 I, LC3 II, fibronectin, and caspase-3 in cellular were determined by western blotting. (d) Quantification of protein levels. Results are expressed as mean SEM. ^#^*p* < 0.05 versus control; ^*∗*^*p* < 0.05 and ^*∗∗*^*p* < 0.01 versus TGF-*β*1 only.

**Figure 2:** DSS reduced FN secretion and apoptosis of NRK-52E cells induced by TGF-*β*1. NRK-52E cells were treated, respectively, with TGF-*β*1(5 ng/ml), DSS (0.8 mg/ml) + TGF-*β*1(5 ng/ml), and rapamycin (10 nM) + TGF-*β*1(5 ng/ml) for 48 h (*n* = 3, per group). (a) Protein levels of fibronectin and caspase-3 in cellular were determined by western blotting. (b) Quantification of protein levels. Results are expressed as mean SEM. ^#^*p* < 0.05 versus control; ^*∗*^*p* < 0.05 versus TGF-*β*1 only.

**Figure 3:** DSS promoted autophagy of NRK-52E cells induced by TGF-*β*1. NRK-52 E cells were treated with TGF-*β*1(5 ng/ml), DSS (0.8 mg/ml) + TGF-*β*1(5 ng/ml), and rapamycin (10 nM) + TGF-*β*1(5 ng/ml), respectively, for 48 h (*n* = 3, per group). (a) Cellular protein levels of LC3 I, LC3 II, Beclin 1, p-mTOR, mTOR, and p62 were determined by western blotting. (b) Quantitative comparison of protein levels. (c) Immunofluorescence images of the LC3B expression. (d) The average fluorescence density of each group was calculated. Results are expressed as mean SEM. ^#^*p* < 0.05 versus control; ^*∗*^*p* < 0.05 and ^*∗∗*^*p* < 0.01 versus TGF-*β*1 only.

**Figure 4:** DSS can suppress the autophagy inhibition of 3-MA. NRK-52 E cells were starved for 24 h and then treated with 3-MA (10 mM) and 3-MA (10 mM) + DSS (0.8 mg/ml) for another 24 h (*n* = 3, per group).(a) Cellular protein levels of LC3 I, LC3 II, Beclin 1, p-mTOR, and mTOR were determined by western blotting. (b) Quantitative comparison of protein levels. (c) Immunofluorescence images of LC3B expression. (d) The average fluorescence density of each group was calculated. Results are expressed as mean SEM. ^#^*p* < 0.05 versus control; ^*∗*^*p* < 0.05 and ^*∗∗*^*p* < 0.01 versus 3-MA only.

**Table 1:** Danggui Shaoyao San components.

Chinese term	Generic name	Scientific name	Product lot
Danggui	*Angelica sinensis* (Oliv.) Diels	*Angelicae sinensis radix*	201103
Baishao	*Paeonia lactifora* Pall.	*Paeoniae radix alba*	20200925-1
Chuanxiong	*Ligusticum chuanxiong* Hort.	*Chuanxiong rhizoma*	201109
Fuling	*Poria cocos* (Schw.) Wolf	*Poria*	201117
Baizhu	*Atractylodes macrocephala* Koidz.	*Atractylodis macrocephalae rhizoma*	20201016-1
Zexie	*Alisma orientale* (Sam.) Juzep.	*Alismatis rhizoma*	201024

## Data Availability

The data used to support the findings of this study are available from the corresponding author upon request.
